# Application Value of Nutrition Support Team in Chemotherapy Period of Colon Cancer Based on Internet Multidisciplinary Treatment Mode

**DOI:** 10.1155/2022/8234769

**Published:** 2022-07-23

**Authors:** Jianfeng Chen, Bo Wang, Xiaobin Yin, Qifei Liang, Yucheng Li, Xingjiang Xie, Xuehui Zeng

**Affiliations:** Gastrointestinal Surgery, People's Hospital of Wenjiang District, 611130 Chengdu City, Sichuan Province, China

## Abstract

**Objective:**

To explore the application value of the nutrition support team in chemotherapy period of colon cancer based on the internet multidisciplinary treatment mode.

**Methods:**

For the method of retrospective study, 90 patients with colon cancer admitted to our hospital from August 2018 to August 2020 were selected as the study subjects. They were equally divided into the experimental group (*n* = 45) and the control group (*n* = 45) according to the order of initials and the method of parity group. The control group was given conventional nutrition support, and the experimental group was given the nutrition support under the internet multidisciplinary treatment mode. The serum tumor marker levels (CEA and CA19-9), immune function indexes, nutrition indicators, and the incidence of adverse reactions were compared between the two groups before and after intervention.

**Results:**

The serum tumor marker levels in the experimental group after intervention were significantly lower than those in the control group (*P* < 0.001). The immune function indexes in the experimental group after intervention were significantly better than those in the control group (*P* < 0.001). The nutrition indicators in the experimental group after intervention were significantly better than those in the control group (*P* < 0.001). The incidence of gastrointestinal adverse reactions above grade 2 in the experimental group was significantly lower than that in the control group (*P* < 0.05). There were 20 patients with myelosuppression, 2 patients with neurotoxicity, and 1 patient with hand and foot syndrome in the experimental group, while 22 patients with myelosuppression, 4 patients with neurotoxicity, and 2 patients with hand and foot syndrome in the control group, with no significant difference in the incidence of adverse reactions between the two groups (*P* > 0.05).

**Conclusion:**

The nutrition support team under the internet multidisciplinary treatment mode can improve the immune function of chemotherapy patients with colon cancer and enhance their nutritional level, thereby reducing the incidence of adverse reactions and improving the chemotherapy effects.

## 1. Introduction

Colon cancer is a malignant tumor originating from epithelial cells of colon mucosa, and the incidence rate has shown an upward trend in recent years, with the incidence rate of 0.3‰ [1]. Surgery and chemotherapy are the focus of comprehensive treatment programs. For colon cancer patients with radical resection, the application of adjuvant chemotherapy before or after surgery can improve the 3-year recurrence-free survival of patients and reduce the possibility of metastasis [2, 3]. For colon cancer patients who cannot be treated surgically, chemotherapy reduces the lesions, which allows patients to regain the opportunity for surgery. Therefore, chemotherapy is recommended as the core treatment measure for patients with colon cancer in the guidelines of the National Comprehensive Cancer Network (NCCN) [4]. In recent years, the practice has gradually confirmed that adjuvant chemotherapy improves the median survival period of colon cancer patients, and the patients with liver metastasis benefit more especially [5]. However, patients with colon cancer often have multiple diseases before chemotherapy, and the incidence of malnutrition is about 40.0% [6]. Long-term or short-term chemotherapy can cause adverse reactions such as nausea, vomiting, and myelosuppression, which further affects the uptake rate of nutrients. If patients with intestinal obstruction have a poor dietetic level before chemotherapy, severe malnutrition will be more likely to occur during chemotherapy, and the immunosuppression will be more obvious [7]. Patients with colon cancer are more prone to anemia due to the malnutrition, thereby reducing the level of plasma protein, which affects the absorption, metabolism, and excretion of chemotherapy drugs. The incremental drug toxicity reduces the number of chemotherapy, and some patients even give up chemotherapy completely [8]. Scholars Kaška et al. have found that the survival period of patients with low body mass treated by comprehensive therapy is significantly shortened, confirming that nutritional status can affect the prognosis of patients with chemotherapy and surgery [9]. Therefore, it is crucial for patients with colon cancer to receive nutrition support during chemotherapy.

NCCN has proposed that patients with colon cancer need multidisciplinary treatment during chemotherapy to closely assess their condition changes [10]. Multidisciplinary treatment (MDT) means that the medical staff coming from different subjects provide patients with independent suggestions about diagnosis and treatment, implement efficient medical services, and formulate the best treatment plans with individual differences according to patients' condition based on the support of data system. In 2016, the National Family Planning Commission in China pointed out that the oncology department should actively implement the treatment mode of single disease and multiple subjects [11]. However, the plan of nutrition support team under the MDT mode has not been implemented due to the practical factors. In recent years, with the continuous development of smart healthcare, the experience accumulated by internet diagnosis and treatment has provided a better reference model for the development of MDT. In particular, big data of medical has become an important data source for MDT. In the internet MDT mode, the working efficiency of the nutrition support team may be significantly improved, which is conducive to improving the effect of nutrition support in patients with colon cancer during chemotherapy. In the internet MDT mode, the work efficiency of the nutrition support team may be significantly improved, which is conducive to improving the nutrition support effect of patients with colon cancer during chemotherapy. Based on this, this study explored the application value of nutrition support team in the chemotherapy period of colon cancer under the internet MDT mode.

## 2. Materials and Methods

### 2.1. Research Design

The retrospective study was conducted in our hospital from August 2018 to August 2020. The study subjects and researchers did not understand the grouping of this experiment, and the research designers were responsible for arranging and controlling the experiment.

### 2.2. Inclusion and Exclusion Criteria

Inclusion criteria: (1) The patients were diagnosed with colon cancer by colonoscopy, which met the diagnostic criteria in the Guidelines for the Diagnosis and Treatment of Colon Cancer [12], and they were diagnosed and treated with interventional therapy for the first time. (2) Patients had definite clinical stages and had indications for chemotherapy. (3) Patients had no abnormal immune function before chemotherapy. (4) Patients were expected to survive more than 3 months. (5) Patients had no history of long-term fasting. (6) Patients could cooperate with the comprehensive therapeutic strategies in the MDT mode. Exclusion criteria are as follows: (1) patients with metastasis in vitals such as abdominal cavity and liver, (2) patients with dysfunction in vitals, (3) patients with the second primary tumor, (4) patients with the contraindication of chemotherapy, (5) patients with the contraindication of nutrition support, (6) patients with language dysfunction and who could not communicate with others, (7) patients with low immune function before chemotherapy and poor tolerance to chemotherapy, and (8) patients with endocrine system diseases

### 2.3. General Information

In the study, 90 patients were equally divided into the experimental group (*n* = 45) and the control group (*n* = 45) according to the order of initials and the method of parity group. On the day when the patients agreed to participate in the study, the study group collected the data of sociodemography and clinical manifestation. It was found that there was no statistical difference in the patients' general information between the two groups by comparison (*P* > 0.05), which was comparable. In the experimental group, there were 25 males and 20 females with an average age of 51.27 ± 5.20 years old. Before intervention, the body weight was 55.65 ± 2.65 kg, the BMI was 21.22 ± 1.23 kg/m^2^, and the ECOG score was 0.67 ± 0.60 points. In Dukes staging, grade A had 2 cases, grade B had 18 cases, grade C had 18 cases, and grade D had 7 cases. There were 8 cases with hypertension, 6 cases with diabetes mellitus, and 15 cases with intestinal obstruction. In the control group, there were 26 males and 19 females with an average age of 51.22 ± 2.43 years old. Before intervention, the body weight was 55.74 ± 2.40 kg, the BMI was 21.24 ± 1.28 kg/m^2^, and the ECOG score was 0.64 ± 0.60 points. In Dukes staging, grade A had 1 case, grade B had 19 cases, grade C had 19 cases, and grade D had 6 cases. There were 8 cases with hypertension, 7 cases with diabetes mellitus, and 17 cases with intestinal obstruction.

### 2.4. Moral Consideration

This study was in line with the principles of Declaration of Helsinki (2013) [13], and patients signed the informed consent.

### 2.5. Methods

#### 2.5.1. Chemotherapy

Patients in both groups were treated with the FOLFOX4 regimen. On the first day, they received oxaliplatin (Jiangsu Hengrui Pharmaceutical Co., Ltd.; NMPA approval No.: H20050962) by intravenous infusion at a dose of 85 mg/m^2^. On the first and second days, they received calcium leucovorin (New Asiatic Pharmaceutical Co., Ltd.; NMPA approval No.: H20113395) by intravenous infusion at a dose of 200 mg/m^2^ and received 5-fluorouracil (Beijing Zizhu Pharmaceutical Co., Ltd.; NMPA approval No. H11020069) by intravenous infusion at a dose of 400 mg/m^2^. With 14 days as a chemotherapy cycle, two chemotherapy cycles were performed. The measures of symptomatic treatment such as the prevention of vomiting and the protection of stomach were routinely taken before chemotherapy.

#### 2.5.2. Control Group

The control group was given conventional nutrition support. Firstly, patients were given complete parenteral nutrition, with the heat maintained at 30 kcal/kg/d and the energy ratio of lipid emulsion to glucose as 2 : 3. They were given the enteral nutrition gradually, supplemented by nutritional agents with the daily heat supply of 500 kcal. Patients with severe gastrointestinal reactions also received parenteral nutrition until the surgery was performed.

#### 2.5.3. Experimental Group

The experimental group was given the nutrition support under the internet MDT mode. (1) The MDT team about colon cancer was established. The team members included doctors and nursing staff coming from department of medical oncology in alimentary system, colorectal surgery, anesthesia department, intervention department, nutrition department, imaging department, laboratory department, and pharmacy department, and all participants joined the MDT WeChat group. The doctor and nursing teams were divided into the data, administration, and instruction groups. The managers were clinicians and nursing staff with high qualification and rich experience, whose primary responsibilities were to make an induction and summary of the data and monitor the implementation of the team work. The team members needed to deeply understand the MDT mode through the ways of master lectures and evidence-based medicine and fully learn how to formulate the medical decisions based on the data and apply the decisions to medical process. (2) The internet database was established with the help of the hospital diagnosis and treatment platform, which contained the patient data, medical data, nursing data, and literature data. The patient data were primary data mainly including the basic information of patients (name, gender, the duration of hospitalization, etc.), treatment information (attending physicians, surgeons, surgical methods, etc.), economic information (medical expenses), and MDT information (medical process, neoadjuvant therapy, adjuvant therapy, etc.). The medical data included doctors' orders and all kinds of inspection and examination information and patients' data of clinical symptoms and test indicators. The nursing data included doctors' orders and the implementation of inspection and examination, the common clinical scales such as the scale of Hamilton negative emotion and the scale of NRS nutrition risk assessment, and the questionnaire data collected from patients. The literature data included the data from Chinese and foreign professional literature on colon cancer for doctors and nurses to consult. (3) The instruction group established a diagrammatic figure of MDT nutrition support for colon cancer patients according to the data collected from the internet database and divided the work about nutrition support into three stages during chemotherapy. The first stage was the preparation of nutrition support, which is aimed at comprehensively developing the nutrition support strategies combining the mental status, nutritional status, and various clinical indicators to improve the treatment and nursing compliance and meeting the needs of mental and physical health of patients. The second stage was the implementation of nutrition support, which is aimed at improving the patients' immune function, alleviating the adverse reactions of chemotherapy, and providing good support for subsequent treatment by targeted measures of nutrition support. The third stage was from the end of chemotherapy to discharge, which was dominated by collecting feedback from patients to provide health guidance for them. (4) The administration group formulated the flow chart according to the tasks of each stage and supervised the implementation. The data group dynamically collected the internet data at each stage to facilitate the team to evaluate the implementation effects of the nutrition support under the MDT mode at any time. In the instruction group, the chief experts updated the progress once every 3 days, and the doctors and nursing staff made supplements and discussions in the WeChat group with weekly meetings offline. (5) The measures of nutrition support in the experimental group were formulated by the MDT team according to the above steps on the basis of the control group. The nursing navigators accompanied the patients and answered their questions throughout the intervention and delivered messages dynamically and timely between the MDT nutrition support team and the patients.

### 2.6. Observation Indexes

#### 2.6.1. The Serum Tumor Marker Levels

The fasting venous blood was taken from the patients in the morning before and after intervention to measure the levels of CEA and CA19-9 by radioimmunoassay using a Roche electrochemiluminescence analyzer with original matching reagents (NMPA (I) 20113402843) and to measure the CA72-4 level by enzyme-linked immunosorbent assay (Beijing Kewei Clinical Diagnostic Reagent Co., Ltd.; NMPA approval No. S20060028).

#### 2.6.2. Immune Function Indexes

The fasting venous blood was taken in the morning before and after intervention to measure the levels of CD4^+^, CD8^+^, CD4^+^/CD8^+^, Treg, Th9, and Th17 by a flow cytometry (ACEA BIO (Hangzhou) Co., Ltd.; Zhejiang Medical Products Administration Certified No. 20142400581).

#### 2.6.3. Nutrition Indicators

The body weight of the two groups after intervention was recorded. The fasting venous blood of patients in the morning was taken before and after intervention to measure the levels of total protein (TP), albumin (ALB), and hemoglobin (Hb) by an automatic biochemical analyzer with original matching reagents (Sysmex CHEMIX-800 automatic biochemical analyzer, NMPA approval No. 20112403311).

#### 2.6.4. Incidence of Adverse Reactions

The adverse reactions of patients in the two groups during chemotherapy were recorded according to the World Health Organization (WHO) evaluation criteria for adverse reactions to anticancer drugs [14], and the incidence of adverse reactions was calculated.

### 2.7. Statistical Treatment

In this study, the experimental data were processed by SPSS20.0, and GraphPad Prism 7 (GraphPad software, San Diego, USA) was used to draw pictures of the data. The items included in the study were enumeration data and measurement data tested by *χ*^2^ and *t*-test. When *P* < 0.05, the differences were considered to be statistically significant.

## 3. Results

### 3.1. Serum Tumor Marker Levels

The serum tumor marker levels in the experimental group after intervention were significantly lower than those in the control group (*P* < 0.001) (see details in Figure 1).

There was no statistical difference in the levels of CEA, CA19-9, and CA72-4 between the experimental group and the control group before intervention (20.11 ± 1.22 vs. 20.15 ± 1.24, 80.54 ± 2.65 vs. 80.67 ± 2.41, and 23.98 ± 1.25 vs. 23.87 ± 1.20, *P* > 0.05). The levels of CEA, CA19-9, and CA72-4 in the experimental group after intervention were significantly lower than those in the control group (5.67 ± 0.53 vs. 6.44 ± 0.60, 30.55 ± 2.68 vs. 39.68 ± 3.11, and 12.68 ± 1.25 vs. 17.12 ± 1.30, *P* < 0.001).

### 3.2. Immune Function Indexes

The immune function indexes in the experimental group after intervention were significantly better than those in the control group (*P* < 0.001) (see details in Figure 2).

There was no statistical difference in the levels of CD4^+^, CD8^+^, and CD4^+^/CD8^+^ between the experimental group and the control group before intervention (37.52 ± 3.65 vs. 37.60 ± 3.45, 25.98 ± 2.65 vs. 26.05 ± 2.41, and 1.35 ± 0.32 vs. 1.38 ± 0.30, *P* > 0.05). The levels of CD4^+^, CD8^+^, and CD4^+^/CD8^+^ in the experimental group after intervention were significantly better than those in the control group (30.98 ± 3.11 vs. 35.11 ± 3.02, 36.98 ± 2.65 vs. 28.98 ± 3.11, and 08.9 ± 0.12 vs. 1.12 ± 0.23, *P* < 0.001).

There was no statistical difference in the levels of Treg, Th9, and Th17 between the experimental group and the control group before intervention (10.11 ± 0.54 vs. 10.15 ± 0.60, 1.40 ± 0.15 vs. 1.42 ± 0.15, and 5.05 ± 0.35 vs. 5.10 ± 0.36, *P* > 0.05). The levels of Treg, Th9, and Th17 in the experimental group after intervention were significantly better than those in the control group (5.11 ± 0.34 vs. 8.96 ± 0.57, 0.67 ± 0.05 vs. 1.32 ± 0.44, and 2.67 ± 0.24 vs. 3.68 ± 0.30, *P* < 0.001).

### 3.3. Nutrition Indicators

The nutrition indicators in the experimental group after intervention were significantly better than those in the control group (*P* < 0.001) (see details in Figure 3).

There was no statistical difference in body weight and the levels of TP, ALB, and Hb between the experimental group and the control group before intervention (55.65 ± 2.65 vs. 55.74 ± 2.40, 58.62 ± 2.56 vs. 58.67 ± 2.47, 33.65 ± 2.65 vs. 33.24 ± 2.57, and 115.65 ± 2.65 vs. 116.00 ± 2.14, *P* > 0.05). The body weight and the levels of TP, ALB, and Hb in the experimental group after intervention were significantly better than those in the control group (59.55 ± 2.65 vs. 56.65 ± 2.47, 70.12 ± 2.65 vs. 60.55 ± 2.75, 40.65 ± 2.47 vs. 33.84 ± 2.68, and 128.98 ± 5.98 vs. 119.21 ± 4.50, *P* < 0.001).

### 3.4. Incidence of Adverse Reactions

There were gastrointestinal reactions of different degrees during chemotherapy in the two groups. In the experimental group, there were 18 patients with nausea and vomiting, 10 patients with diarrhea, 6 patients with nausea and vomiting above grade 2, and 5 patients with diarrhea above grade 2. There were 26 patients with nausea and vomiting, 18 patients with diarrhea, 15 patients with nausea and vomiting above grade 2, and 13 patients with diarrhea above grade 2 in the control group. The incidence of gastrointestinal adverse reactions above grade 2 in the experimental group was significantly lower than that in the control group (*P* < 0.05). In addition, there were 20 patients with myelosuppression, 2 patients with neurotoxicity, and 1 patient with hand and foot syndrome in the experimental group and 22 patients with myelosuppression, 4 patients with neurotoxicity, and 2 patients with hand and foot syndrome in the control group. There was no significant difference in the incidence of adverse reactions between the two groups (*P* > 0.05).

## 4. Discussion

The incidence rate of colon cancer has increased year by year, and the number of patients who need nutrition support during perioperative period has gradually increased. The combination of chemotherapy and surgery is an important comprehensive treatment program approved by many international guidelines for diagnosis and treatment of colon cancer [15]. The clinical value of chemotherapy (or adjuvant chemotherapy) has been confirmed by many studies in recent years, but this program inevitably needs coordination with other treatment measures such as nutrition support. Scholars Plassmeier et al. have claimed that the incidence of malnutrition in patients with malignant tumors is 39.0%, while the incidence of patients with advanced gastrointestinal cancer is higher [16], and the probability of malnutrition in patients with colon cancer is 40.0–50.0% [17]. More and more reports showed that the nutrition support for patients with malignant tumors during chemotherapy can improve the chemotherapy tolerance and enhance the chemotherapy compliance, thereby improving the chemotherapy effect. Therefore, nutrition support is an indispensable part of the comprehensive treatment programs for colon cancer patients, and it is extremely important to deepen the application exploration of nutrition support under the MDT mode.

The MDT mode means that the medical staff coming from different fields provide treatment programs with individual differences for specific patients, so that patients can obtain the best support for treatment. Previous practice has shown that the MDT mode can realize the integration and sharing of medical resources, improve the accuracy of treatment, and shorten the treatment time of patients [18, 19]. With the support of internet big data, smart medical platform provides more possibilities for the application of the MDT mode in nutrition support. In this study, the targeted nutrition support strategies were formulated based on the data obtained from the hospital diagnosis and treatment platform. The study also found that the personalized nutrition support strategies supported by data could better improve the psychological and physical condition of patients and enhance their compliance of nutrition support. The MDT nutrition support team could dynamically adjust the nutrition support plans of patients by online discussion and offline meeting in the experimental group according to the data feedback, so that patients could obtain better nutrition support. Therefore, the nutrition indicators in the experimental group after intervention were significantly better than those in the control group (*P* < 0.001). Since the decline of immune function is an important manifestation of malnutrition in patients with malignant tumors [20], the immune indexes of patients will be improved with the improvement of nutrition status, so that the immune status of patients in both groups after nutrition support is improved. Under the condition of malnutrition, the immune cells of patients such as Treg, Th9, and Th17 show excessive differentiation, which weakens the kill effect of specific and nonspecific immune response on tumor cells, so that patients cannot inhibit cancer through the immune system. The combination of neoadjuvant chemotherapy and nutrition support can ensure that patients obtain sufficient energy sources to enhance self-defense mechanism and improve the metabolic function of organs, thereby enhancing the targeting of chemotherapy without excessively damaging the normal cells [21]. Scholars Keskin et al. have shown that neoadjuvant chemotherapy and nutrition support can improve the levels of CD4^+^, CD8^+^, and CD4^+^/CD8^+^ in elderly patients with colon cancer [22]. In this study, patients had better improvement in immune function under the internet MDT mode due to the better nutrition indicators in the experimental group.

Nutrition support can maintain the continuity of their gastrointestinal function by improving the immune function and nitrogen balance of colon cancer patients, thereby enhancing the barrier and immune function and accelerating the recovery of intestinal mucosa [23], so that patients in the experimental group were less likely to have gastrointestinal adverse reactions above grade 2. According to Guo, adverse reactions are the important factors affecting patients' willingness and the effect of chemotherapy, and severe toxicity reduces the number of chemotherapy in patients and affects the promotion effect of neoadjuvant chemotherapy for surgery [24]. The reduction of adverse reactions makes patients more willing to accept chemotherapy, and the improvement of immune function also makes them more resistant to the chemotherapy. This study showed that the nutrition support under the internet MDT mode could act on many aspects such as immunity and gastrointestinal function by improving the nutritional indicators to synergistically enhance the chemotherapy effect of patients from different aspects. The performance was that the serum tumor marker levels in the experimental group after intervention were significantly lower than those in the control group (*P* < 0.001). Another study has shown that the MDT mode is able to improve the 5-year survival rate of patients with advanced colorectal cancer [25]. The survival rate of patients was not counted in this study, and the influence of nutrition support under the internet MDT mode on the survival rate of patients with colon cancer needs to be explored and demonstrated further.

## 5. Conclusion

The nutrition support team under the internet multidisciplinary treatment mode can improve the immune function of chemotherapy patients with colon cancer and enhance their nutritional level, thereby reducing the probability of adverse reactions and improving the effect of chemotherapy.

## Figures and Tables

**Figure 1:** Serum tumor marker levels (*x̅*±*s*). (a) CEA level. (b) CA19-9 level. (c) CA72-4 level.

**Figure 2:** Levels of immune function indexes (*x̅*±*s*). (a) Levels of CD4^+^, CD8^+^, and CD4^+^/CD8^+^ before intervention. (b) Levels of CD4^+^, CD8^+^, and CD4^+^/CD8^+^ after intervention. (c) Levels of Treg, Th9, and Th17 before intervention. (d) Levels of Treg, Th9, and Th17 after intervention.

**Figure 3:** Levels of nutrition indicators (*x̅*±*s*). (a) Body weight. (b) TP level. (c) ALB level. (d) Hb level.

## Data Availability

Data to support the findings of this study is available on reasonable request from the corresponding author.
